RETRACTED

# Effect of Rehabilitation Physical Training on PE Teaching Sports Injury under Ultrasonic Examination

**DOI:** 10.1155/2022/1470303

**Published:** 2022-09-17

**Authors:** Wangda Li

**Affiliations:** School of Physical Education, Ankang University, Ankang, Shaanxi 725099, China

## Abstract

In order to solve the problem of the effect of rehabilitation physical training on physical education teaching injury, a method based on ultrasonic examination of rehabilitation physical training on physical education teaching injury effect observation method is proposed. In this method, the ISOMED isokinetic muscle strength test, the body shape test, the balance ability test, the lower limb explosive power test, and other methods are used to evaluate the knee joint of patients systematically, and the specific rehabilitation physical training plan is formulated to achieve the treatment purpose. The experimental results show that after the targeted training, a series of indicators on the affected side increase significantly: the power increases by 45.6%, the force increases by 8.3%, and the speed increases by 38.7%. It is concluded that the muscle strength, shape, balance ability, and lower limb explosive power of patients are significantly improved, which lays a solid foundation for athletes to recover smoothly and achieve good competition results.

## 1. Introduction

Physical training itself is a sport with strong sports intensity and high physical energy consumption. In the actual teaching process, when the training intensity required by teachers is too high, students' physical function is difficult to bear, so it is easy to cause injury. Of course, this is only one reason, and the other reason is that the balance between the exercise intensity and the training amount is not fully grasped. Before students' physical training activities, the first thing teachers should do is to lead students to complete the warm-up activities of sports, so that the muscles of the whole body are in a relaxed state, so as to effectively enhance students' muscle toughness [1]. But, in general, when part of the physical education teachers in colleges and universities lead the students to do exercises or a warm-up, they do not fully play the role of the warm-up activity, which consumes time, but the effect is not good. Because the students' understanding of the importance of a warm-up is not sufficient, in the process of preparing activities, they are perfunctory, eventually leading to the generation of sports injury. Unscientific and nonstandard technical movement is the main cause of sports injury. In the process of physical training activities, students, as the adaptable objects and subjects of training activities, have great individual differences and prominent differences in subjects. Each student's physical quality and learning ability will be different. Therefore, when teachers explain the essentials of technical movements, not all students can fully understand the essential skills taught by teachers, and not all students can use them proficiently and achieve standard movements [2]. For example, the football sport looks simple, but it tests the practitioner's body quality, participation attitude, strain capacity, and psychological state. At the same time, under the influence of external factors, it may also may prevent students from keeping a good state on the pitch, which can lead to a technical foul and collision conditions, thus sports injury problems. There is no absolute relationship between the occurrence of sports injuries and specific sports events, but there are some rules that can be used to refer to avoid more injuries. The main reason for the damage is that in the process of exercise, due to the confrontation between the two sides, there are many quick stops and rapid turns and so on, and these postures will inevitably affect the muscles in the waist and abdomen. Obviously, in order to achieve the effect of fitness, we not only need to rely on exercise but also have the ability to analyze the rules of exercise and nursing knowledge [3]. Only in this way can we detect sports injuries in time and treat them quickly. Through the comparison and analysis of the damage area and the relationship between the sports events, it can be found that the damage area is mainly caused by some common action in the process of movement. As a result, there are some laws between the two factors, namely, certain key action and frequent action may cause damage to the corresponding part of the muscle [4]. For example, the most common injury part in football is the ankle and the related joints used in shooting. The shooting action in basketball, including jumping and running, will cause damage to the ankle and peripheral joints. At the same time, if the strength is too high during the passing, it is easy to tear ligaments and damage the meniscus. In addition, long-term confrontation sports can also cause tissue damage, such as muscle strain.

RETRACTED

## 2. Literature Review

The characteristics of intense confrontation and high intensity of football determine that sports injuries will inevitably occur in college football training and competition. After the occurrence of sports injury, the conventional treatment is usually drug treatment or surgical treatment, reduction of training intensity, or suspension to promote the recovery of athletes, as shown in Figure 1 [5]. However, the above conventional treatment methods and treatment arrangements are mainly aimed at the treatment and rehabilitation strategies of the injury site, but they do not solve the root causes of the injury. In fact, in college football training, many acute injuries and chronic injuries are related to the athletes' own physical deficiency or physical decline, which is also an important reason why many sports injury accidents occur near the end of the training [6]. Injury treatment with medical means alone is helpful for the rehabilitation of injured parts, but it cannot solve the problem of athletes' lack of physical strength [7]. Even because of the reduction of training intensity or suspension during the treatment of rest, physical decline may appear in the athletes. In such a situation, coupled with the root causes of the injury of athletes which have not been solved, after the recovery of injury and reentry to normal training activities, athletes are often prone to recurrent injury problems, thus affecting the health level and sports level of athletes. Rehabilitation physical training is significantly different from the injury treatment by medical means alone [8]. Rehabilitation physical training is based on the support of rehabilitation medicine, which organically combines the athlete's rehabilitation and physical training. It not only helps in the treatment and rehabilitation of sports injuries but also can improve the physical reserves of athletes through long-term targeted application in athletes' daily training. This prevents the recurrence of sports injuries and achieves the “1 + 1 > 2” effect of rehabilitation and physical training, allowing athletes to better adapt to the needs of special football training and competitive competitions. Football players not only need sufficient strength qualities but also have higher requirements for qualities such as speed, agility, coordination, and endurance. At the same time, in football, the movements of the lower limbs account for a large proportion. The most common football injury is found to be the knee meniscus injury (prevalence 12.1%) [9]. Because the knee joint is located in the middle of the lower extremity, it needs to bear more stress and performs long-lasting three-dimensional movement, so the probability of injury is greater [10]. In the research, the concept and the method of rehabilitation physical training are applied to patients with knee joint injury, and the systematic and phased assessment is conducted through isokinetic muscle strength, lower limb circumference, and balance ability test methods [11]. According to the test results, the specific rehabilitation physical training can make their knee joints recover well, improve their physical quality and ability, and lay a solid foundation for good competition results.

RETRACTED

## 3. Methods

### 3.1. Retrospective Research Subjects

The patient is female, 18 years old, a Chinese youth female football player, and a defender. During the training of the national team, there was discomfort in the right knee joint, with functional dysfunction and edema in the knee joint. Results of MRI film evaluation by a third-grade hospital are as follows: (1) anterior cruciate ligament (ACL) fracture of the right knee, (2) massive effusion of the right knee joint, and (3) rupture of the medial meniscus of the right knee and atrophy of the quadriceps muscle [12]. The medial meniscus of the right knee was removed, and the anterior cruciate ligament reconstruction of the right knee was performed. And then, physical training is carried out for rehabilitation.

### 3.2. Test Instrument and Method

The ISOMED isokinetic test system (including dynamic instrument, force measurement platform, and computer and various joint test accessories) is used to test isokinetic force. The system can set the movement speed of 0~500°/s. Four movements of knee flexion and extension, knee internal and external rotation, and ankle dorsiflexion/plantarflexion are selected. The slow peak torque is selected as the evaluation index reflecting the maximum muscle strength of the knee and ankle joints of athletes [13]. The body shape test includes body composition and lower limb muscle circumference test. The InBody 3.0 body composition analyzer is used for the comprehensive analysis of human composition. For lower limb circumference, thigh circumference and calf circumference are used to reflect the growth of muscle volume. The balance ability reflects the stability of lower limbs by standing on one foot with eyes closed. Lower limb explosive force is tested by the CMJ mode of a single-leg Counter Movement Jump, and the data are collected by the MYOTEST explosive force tester [14].

### 3.3. Rehabilitation Training Program

According to the patient's injury response and test results, a personalized training program is developed, which is divided into three stages for 5 weeks. The training program is optimized by evaluating the training effect of each stage, so as to ensure the quality of rehabilitation training for patients [15]. See Table 1 for specific training programs.

## 4. Results and Analysis

### 4.1. Isokinetic Muscle Force Test and Analysis

As can be seen from Table 2, the strength of the bilateral knee extensor muscle is significantly different, reaching 18.6%, indicating that the strength of the right quadriceps muscle is weaker than that of the left side. The strength of the bilateral internal pronator muscle group is lower than that of the external pronator muscle group, but the strength of the right internal pronator muscle group is significantly different from that of the left side, reaching 18.2%. The results show that the semitendinosus semimembrane muscle group on the right side of the patient is weaker than that on the left side, and the difference between pronation and supination is large, indicating that the semitendinosus semimembrane muscle on the right side is weaker than the biceps femoris muscle. Bilateral differences in dorsiflexion and plantar flexion are -20% and 18.2%, respectively, indicating that the right dorsiflexor muscle group is stronger than the left side, while the calf triceps is weaker than the left side [16]. Quadriceps atrophy and loss of strength of the medial rotator muscles are caused by the right knee that has undergone ACL reassignment and medial meniscectomy. Due to the lack of knee strength, ankle involvement is increased to maintain lower limb balance, resulting in the right dorsiflexor muscle group being stronger than the left.

RETRACTED

As can be seen from Table 3, the increased range of knee flexion, extension, and ankle joint plantar flexion is obvious, which is directly related to the injury type, injury response, and rehabilitation training arrangement of patients. If the patient suffers from quadriceps atrophy and poor muscle strength, and the quadriceps muscle is the main extensor muscle group, the strength of the quadriceps muscle group can be increased by activating the quadriceps muscle and increasing the strength exercise of the knee extensor muscle group [17]. At the same time, the movement ability of football players on the field requires the plantar-flexion strength of the ankle joint, and the triceps muscle of the calf plays an important role in maintaining the balance of lower limbs and human body upright. In view of this situation, the plantar-flexion strength exercise of the ankle joint is added in training to increase the plantar-flexion strength [18]. Therefore, according to the situation of the muscle strength of the affected side of the athletes, the development of a highly targeted rehabilitation training plan has an obvious effect on the muscle strength recovery of the muscle group of the posterior shoulder joint.

### 4.2. Body Shape Test and Analysis

Table 4 shows that the patient's body weight and muscle weight are significantly changed, with an increase of 1.5 kg and 2.0 kg, respectively. Body weight and muscle weight are improved when the body fat ratio decreases, indicating that the muscle-building training program for patients has achieved certain results [19]. The combination component test shows that the lower limb muscle volume of patients increases, indicating that reasonable rehabilitation training plan has significant effect on the increase of lower limb muscle volume.

RETRACTED

### 4.3. Test and Analysis of Balance Ability and Lower Limb Explosive Force

As can be seen from Table 5, the balance ability of the left and right sides has been strengthened, increasing by 35 s and 50s, respectively. Although the improvement range is large, there is still a certain gap between the balance ability of the affected side and that of the healthy side, and the risk of injury of the affected side is still high in the process of stable support.  Figure 2 shows that explosive power test indexes on the affected side increased significantly after training, with power increasing by 45.6%, force value increasing by 8.3%, and speed increasing by 38.7%, while the healthy side does not increase significantly [20]. At the same time, the explosive force index of the affected side is different from that of the healthy side, and all the data are higher than that of the left side.

## 5. Conclusions

In the research, the observation of the effect of rehabilitation physical training under ultrasonic examination on sports teaching injury is put forward. By using the concept of rehabilitation physical training, athletes' body shape, muscle strength level, explosive power, and balance ability can be improved effectively. By using the testing methods of body shape, function, and muscle strength, athletes can be effectively evaluated before training, monitored during training, and evaluated after training, which can ensure the systematic, effective, and scientific rehabilitation physical training. Rehabilitation physical training is of great significance in the prevention and treatment of sports injury in football projects. The understanding should be strengthened, and the rehabilitation thought centered on treatment should be changed, so as to establish the modern rehabilitation physical training concept of prevention first, treatment second, and prevention and treatment equally.

## Figures and Tables

**Figure 1:** First aid method for sports injury.

**Figure 2:** The increase of the affected side of the explosive power test index after the training.

**Table 1:** Rehabilitation training arrangement.

The training phase	Purpose of training	Training time and schedule	Training content and specific arrangements
Weeks 1-2	Restore knee joint function; improve the basic strength of the affected knee joint	Monday to Friday	(1) Functional training: it involves the movement patterns in the sagittal, coronal, and horizontal planes of the shoulder joint, mainly based on resistance training; the equipment is an elastic band, medicine ball, Swiss ball, etc., 3 sets. Practice moves such as ball squats, lunges, medicine ball standing, and more. (2) Basic strength training: resistance training based on single plane action mode, involving quadriceps femoris, biceps femoris, semimembranosus, triceps calf, etc.; the number of times is 8-12 times; and the number of sets is 3-4 sets.
Weeks 3-4	Knee muscle volume: knee muscle strength	Monday to Friday	Training to increase the volume and strength of the muscles around the knee joint: the resistance training is mainly based on the single-plane movement mode, involving the quadriceps femoris, biceps femoris, semimembranosus, and triceps calf. The equipment is barbell and dumbbell, kettlebell, MIHA, and Technogym multifunctional training equipment; the number of times is 4-8; and the number of groups is 4-6. Practice movements such as sitting knee extension and supine leg hook.
Week 5	Overall strength and endurance of lower body: explosive power of knee joint, special strength	Monday, Wednesday, Friday	(1) The overall strength and endurance of the knee joint: the resistance training is mainly based on the multiplane movement mode. The equipment is Technogym multifunctional training equipment, MIHA centrifugal training equipment, dumbbells, barbells, kettlebells, etc. The number of times is 10-15, and the number of sets is 3-4 groups. Practice movements such as weight-bearing half-squats, multidirectional lunges, and walking with bows and arrows. (2) Knee explosive power and special strength: focus on special movement, jumping, starting, and braking modes and choose elastic bands, medicine balls, etc. for equipment, 10-15 times, and 3-4 groups. Practice movements such as step jumps, court starting, and braking exercises.

RETRACTED

**Table 2:** Isokinetic (60°/s) muscle strength test results of patients before rehabilitation training.

Test indicators		Knee flexion and extension			Internal and external rotation of the knee			Ankle dorsiflexion, plantar flexion		
		Flexion	Extension	Difference	Internal rotation	External rotation	Difference	Dorsiflexion	Plantar flexion	Difference
Peak torque (Nm)	Left	81	150	54.1	22	24	8.3	25	66	62.1
	Right (afflicted)	72	118	61.4	18	22	18.2	30	54	44.4
	Two-sided difference (%)	8.6	18.6	/	18.2	8.3	/	-20	18.2	/

Note: bilateral difference = (left − right)/left × 100%, difference in flexion and extension = (extension − flexion)/extension × 100%, difference in internal and external rotation = (external rotation − internal rotation)/external rotation × 100%, difference in dorsiflexion and plantarflexion = (plantar − dorsiflexion)/plantarflexion × 100%.

**Table 3:** Isokinetic (60°/s) muscle strength test results on the affected side of the patient after rehabilitation training.

Test indicators	Test time	Knee flexion and extension			Internal and external rotation of the knee			Ankle dorsiflexion, plantar flexion		
		Flexion	Extension	Difference	Internal rotation	External rotation	Difference	Dorsiflexion	Plantar flexion	Difference
Peak torque (Nm)	2012.9.24	72	118	61.4	18	22	18.2	30	54	44.4
	2012.10.31	85	142	60	19	24	20.8	28	81	65.4
	Change rate (%)	18.1	20.3	—	5.6	9.1	—	-6.7	50	—

Note: change rate = (poster − anterior)/anterior × 100%, difference in flexion and extension = (extension − flexion)/extension × 100%, difference in internal and external rotation = (external rotation − internal rotation)/external rotation × 100%, difference in dorsiflexion and plantarflexion = (plantar − dorsiflexion)/plantarflexion × 100%.

**Table 4:** Changes in body shape.

Test date	Body composition			Thigh and calf muscle circumference (cm)					
	Weight (kg)	Muscle weight (kg)	Body fat ratio	Thigh root		Knee edge		Calf circumference	
				Left	Right	Left	Right	Left	Right
9.24	52.3	40.3	18.2%	51.5	51.5	37.5	36.5	34.0	34.0
10.31	53.8	42.3	16.6%	51.8	51.6	38.0	37.5	34.3	34.2

**Table 5:** The test changes of balance ability and explosive force.

Test content	Balance ability		Explosive force								
			Power (w/kg)			Force (N/kg)			Speed (cm/s)		
	Left	Right	Left	Right	Difference	Left	Right	Difference	Left	Right	Difference
9.24	70	15	18.8	14.7	29.3	16.7	12.8	30.5	136	106	28.3
10. 31	105	65	19.2	21.4	-10.3	16.9	17.7	-4.5	137	147	-6.8
Change rate (%)	50	266.7	2.1	45.6	—	1.2	38.3	—	0.7	38.7	—

Note: change rate = (back − front)/front × 100%; bilateral difference (%) = (left − right)/right × 100%.

## Data Availability

The data used to support the findings of this study are available from the corresponding author upon request.
